# Vinpocetine and Pyritinol: A New Model for Blood Rheological Modulation in Cerebrovascular Disorders—A Randomized Controlled Clinical Study

**DOI:** 10.1155/2014/324307

**Published:** 2014-12-07

**Authors:** Hayder M. Alkuraishy, Ali I. Al-Gareeb, Ali K. Albuhadilly

**Affiliations:** ^1^Department of Pharmacology, Toxicology and Medicine, College of Medicine, Al-Mustansiriya University, P.O. Box 14132, Baghdad, Iraq; ^2^Department of Pharmacology and Medicine, College of Medicine, Al-Mustansiriya University, P.O. Box 14132, Baghdad, Iraq

## Abstract

Blood and plasma viscosity are the major factors affecting blood flow and normal circulation. Whole blood viscosity is mainly affected by plasma viscosity, red blood cell deformability/aggregation and hematocrit, and other physiological factors. Thirty patients (twenty males + ten females) with age range 50–65 years, normotensive with history of cerebrovascular disorders, were selected according to the American Heart Stroke Association. Blood viscosity and other rheological parameters were measured after two-day abstinence from any medications. Dual effects of vinpocetine and pyritinol exhibit significant effects on all hemorheological parameters (P < 0.05), especially on low shear whole blood viscosity (*P* < 0.01), but they produced insignificant effects on total serum protein and high shear whole blood viscosity (*P* > 0.05). Therefore, joint effects of vinpocetine and pyritinol improve blood and plasma viscosity in patients with cerebrovascular disorders.

## 1. Introduction

Blood and plasma viscosity are the major factors affecting blood flow and normal circulation, so the whole blood viscosity is chiefly affected by plasma viscosity, red blood cell deformability, hematocrit, and other physiological factors. Moreover, increase in the blood viscosity was associated with development of multiple disorders via damaging the vascular endothelium; thus, there is a positive correlation between blood viscosity and cerebrovascular disorders [1].

Plasma viscosity has Newtonian fluid properties and depends mainly on plasma protein, while blood viscosity has non-Newtonian fluid property and depends primarily on red cell deformability and hematocrit [2].

Consequently, blood viscosity is considerably higher in patients with cerebrovascular disorders due to higher hematocrit and also development of atherosclerosis caused by hyperviscosity; thus, unusual raise in blood viscosity was linked to progression of vascular complications; moreover, high blood viscosity correlated with infarct size and augment of the risk of mortality [3, 4]. Furthermore, increase in the blood viscosity induces endothelial damage, inflammation, vascular wall hypertrophy, platelet aggregation, and deterioration in the blood vessels shear stress; all these factors increase risks of stroke and cardiac ischemia [5].

Therefore, whole blood viscosity was regarded as acute phase marker expecting cardiac and cerebral disorders, so blood and plasma viscosity are a rapid simple test to predict the occurrences of disease and thus, a rapid elevation of blood viscosity was connected with twofold increase in death risk [6].

Vinpocetine (ethylapovincaminate) derived from* Vinca minor* and periwinkle leaves has been extensively used in the management of cerebrovascular disorders via increase in cerebral blood flow, neuroprotection, and improvement of memory functions [7]. Specifically, vinpocetine acts via the following mechanisms [8–11]:

- blocking voltage sensitive Na^+^ channels leading to intracellular decreasing of Na^+^ and Ca^+^ ions which are responsible for ischemic induced excitotoxicity;
- inhibition of cGMP phosphodiesterase and thus increase of cGMP in vascular endothelium causing vasodilation;
- activation of peripheral benzodiazepine receptors which are involved in neuroprotection;
- anti-inflammation and antioxidation, thus preventing rise in blood viscosity;
- modulation of mitochondrial transition pore leading to cardiovascular protection;
- protection from glutamate-induced neurotoxicity.

All these mechanisms of vinpocetine pointed to the protection effects of vinpocetine that are used in prevention of vascular disorders caused via blood and plasma hyperviscosity; also vinpocetine improves brain perfusion through cerebral vasodilation without affecting the cardiovascular resistance; thus, it prevents deleterious neurotoxic effect of hyperviscosity [12].

Also, cGMP reduced in erythrocyte during hyperviscosity; thus, cGMP induced by vinpocetine in addition to vasodilator effect might modulate blood viscosity [13].

Pyritinol is an analogue to pyridoxine but does not produce any action of pyridoxine; it is nootropic via unknown mechanism, but it exerts several effects [14–16]:

- augmentation of cerebral cholinergic system, thus improving memory function;
- antioxidant effect and potent free radical scavenger, thus preventing development of blood viscosity;
- vasodilator and improving of cellular glucose metabolism;
- enhancing of white blood cell survival and migration;
- prevention of cell membrane protein polymerization, especially neuronal and erythrocyte membranes.

Because of these findings, our hypothesis was that the vinpocetine and/or pyritinol improve blood viscosity; therefore, the aim of the present study is to evaluate the effect of vinpocetine and/or pyritinol on blood viscosity.

## 2. Patients and Methods

The present study was accomplished in Al-Mustansiriya University, College of Medicine, Departments of Pharmacology and Internal Medicine, in cooperation with Clinical Laboratory Unit in Al-Yarmouk Teaching Hospital, Bagdad, Iraq, during March of 2014. The clinical study was permitted via confined logical scientific team foundation. Thirty patients (twenty males + ten females) with age range 50–65 years, normotensive with history of cerebrovascular disorders, were selected according to the American Heart Stroke Association Diagnostic Criteria [17] for this clinical study; sixteen of them were smokers and diabetics. Blood viscosity and other rheological parameters were measured after two-day abstinence from any medications except antidiabetic agents. Then the patients were divided into three groups:

Group A: ten patients take vinpocetine 10 mg/day;

Group B: ten patients take pyritinol 100 mg/day;

Group C: ten patients take vinpocetine 10 mg plus pyritinol 100 mg daily.

After two weeks of therapy 10 mL venous blood was taken for measurement of blood viscosity and other parameters. These are the following:

 hematocrit measurement: HCT haematocrit regarded as the red material in blood HCT g/L measured by microhematocrit tube at 10000/minutes RPM for five minutes [18];
 total serum protein (TP) g/dL measured by automated analyzer (Nephstar Plus three-channel protein analyzer, Yima Opto-Electrical Technology Co. Ltd.) [19];
 serum fibrinogen measured by Fibrinogen Human ELISA Kit (ab108841) [20];
 measurement of blood viscosity, whole blood viscosity (WBV) [21–24]: measured by capillary viscometer (0.9 mm diameter, 51720/111 Schott-Gerate type) in relation to distilled water viscosity;
 relative viscosity = flow time of blood (sec)/flow time of D.W sec;
 actual viscosity = relative viscosity − D.W viscosity;
 D.W viscosity = 0.9615 cP;
 high shear rate: WBV = (0.12 × HCT%) + 0.17(TPg/dL−2.07);
 low shear rate: WBV = (1.89 × HCT%) + 3.76(TPg/L−78.42);
 kinematic viscosity (*v*) = actual blood viscosity (*η*)/blood density (*p*)[25, 26];
 blood density = 1.060 kg/m^3^ at 37°C;
 kinematic viscosity: fluid viscosity without force references;
 RBC rigidity index (RRI) = blood viscosity/plasma viscosity [27];
 plasma viscosity measured by low shear 30 viscometers at shear rate of 69.5 s^−1^ (automated viscometer);

drugs used in this clinical study: vinpocetine (cavinton tablet 10 mg, ASIA Pharmaceutical Industries) and pyritinol (encephabol tablet 100 mg, Merck KGaA & Co Werk Spittal, Hosslglasse 9800 Spittal/Drau, Austria);

 statistical evaluation and significance between the different groups: done via using Student's *t*-test when the *P* value was less than 0.05, and the data were expressed as mean ± SD.

## 3. Results

Vinpocetine significantly improves the serum fibrinogen, blood viscosity, plasma viscosity, kinematic viscosity, and erythrocyte rigidity index (*P* < 0.05), but it produced highly significant effect on low shear whole blood viscosity (*P* < 0.01), while vinpocetine effects on hematocrit, total serum protein, and high shear whole blood viscosity were insignificant in comparison with pretreatment values (*P* > 0.05, Table 1).

Pyritinol oral therapy 100 mg/day for two weeks showed significant effects on blood viscosity and plasma viscosity (*P* < 0.05) and highly significant effect on the low shear whole blood viscosity, while it produced insignificant effects on other rheological parameters (*P* > 0.05, Table 2).

Joint effects of vinpocetine and pyritinol (vinpocetine 10 mg/day plus pyritinol 100 mg/day) were shown on all hemorheological parameters (*P* < 0.05), especially on low shear whole blood viscosity (*P* < 0.01), but there are insignificant effects on total serum protein and high shear whole blood viscosity (*P* > 0.05, Table 3).

Regarding the gender differences in RRI (red blood cell rigidity index), in males (number 20) and females (number 10), there are differences in gender response to vinpocetine and/or pyritinol therapy, but this difference in RRI did not reach the level of significance (*P* < 0.05), except the combined vinpocetine and pyritinol which showed significant effect (*P* < 0.05, Figure 1).

## 4. Discussion

The significance of blood rheological factors like whole blood viscosity, erythrocyte sedimentation, erythrocyte deformability, fibrinogen, and hematocrit in the progression of cerebrovascular damage has been established and thus elevation of hemorheological parameters caused cerebral hypoperfusion via blighted brain microcirculation [28]. Elevation in whole blood viscosity decreases blood flow and causes vascular occlusions; also, red blood cells form 99% of all blood cells and they are normally deformable which allows them to adapt during different circulation conditions, but when erythrocyte turns into nondeformable status the whole blood viscosity elevates [29, 30].

Commencing this universal explanation it will be apparent that the erythrocyte and hematocrit are principal regulators and determinants of whole blood viscosity; also low shear whole blood viscosity is related to erythrocyte deformability, while high shear whole blood viscosity is proportionally related to the hematocrit and fibrinogen levels [31]; this may explain the highly significant effects of vinpocetine and/or pyritinol on reduction of low shear whole blood viscosity via enhancement of erythrocyte deformability, regarding the high shear whole blood viscosity; vinpocetine but not pyritinol decreases fibrinogen without affecting hematocrit; therefore vinpocetine and pyritinol have shown insignificant effects on high shear blood viscosity when they were used alone or in combination which might be due to inability of any one of them to reduce hematocrit.

This study showed that vinpocetine significantly improves the blood viscosity at low shear type, reduced fibrinogen level, and improves kinematic viscosity and erythrocyte rigidity. All these effects lead to the augmentation of cerebral blood flow and increase in brain perfusion and oxygen supply in normal healthy cerebral area and around ischemic area in stroke patients; these effects are mainly related to the reduction in whole blood viscosity and induction of erythrocyte deformability.

The mechanical stress as in atherosclerosis and inflammatory conditions causes an increase in the ca^+^ entry into erythrocyte leading to reduction in deformability property of erythrocyte; this leads to elevating the blood viscosity; since vinpocetine inhibits Na^+^-dependent Ca^+^ channels at erythrocyte membrane like the effect of verapamil, vinpocetine enhances the erythrocyte deformability. Moreover, erythrocytes deformability was linked via stimulation of cGMP pathway which was augmented by vinpocetine [32].

Furthermore, drugs that inhibit the phosphodiesterase enzyme (PDE) like pentoxifylline improve blood viscosity via amelioration of erythrocyte deformability; thus vinpocetine reduced the erythrocytes aggregations through cGMP-dependent pathway leading to the improvement in erythrocyte deformability [33].

Muravyov et al.'s 2011 study showed that the administration of pentoxifylline for four-week duration of therapy improves the blood viscosity via activation of phosphodiesterase pathway like the effect of vinpocetine [34].

Moreover, vinpocetine is regarded as antioxidant via free radical scavenger and inhibition of membrane lipid peroxidation of erythrocyte; also, statins and other antioxidants like vinpocetine improve erythrocytes deformability and ameliorate the central and peripheral hemorheological properties [35, 36]; thus antioxidant effect of vinpocetine may produce a potential effect in reduction of blood viscosity.

It is well known that fibrinogen elevates blood flow resistance at microcirculation; as a result the non-Newtonian property of blood will reduce causing elevation in the blood viscosity and decrease in the blood flow; in spite of collateral circulation being frequently present, the oxygen supply and extraction are blighted also; fibrinogen increases risk of viscosity-induced thromboembolic disorders which was resistant to anticoagulant action; also anticoagulant is ineffective in reduction or amelioration of hyperviscosity [37].

Blood viscosity was higher at morning; this circadian rhythm is due to higher fibrinogen level at morning which explained the higher rate of stroke at morning [38]; this also explained why we do this study at morning to evaluate the maximum level of blood viscosity and evaluate the higher potential effects of vinpocetine and pyritinol.

Chronic diabetic hyperglycemia inhibits erythrocyte membrane protein kinase leading to loss of erythrocyte deformability causing diabetic vascular complications and elevation in the blood viscosity; also high blood glucose seen in diabetes mellitus is identified to have a harmful consequence on red blood cells arrangement and rheological uniqueness, which were ultimately donated for diabetic complications [39].

Moreover, diabetes-induced hyperglycemia causes reduction in plasma PH, and this reduction in PH leads to increase in the erythrocyte rigidity; therefore, it was proposed that the erythrocyte rigidity augmented chiefly via hyperglycemia and acidity, thus increasing erythrocyte trapping and rising in blood flow resistance which per se elevates the blood viscosity [40]. Therefore, in the present study approximately half of the patients were diabetic and both vinpocetine and pyritinol improve blood viscosity via improving erythrocyte deformability, so vinpocetine or pyritinol may be of significance in reduction of diabetes-induced hyperviscosity and improvement of erythrocyte deformability derangements.

Gender differences in blood viscosity related to the erythrocyte rigidity and aging. There are major dissimilarities among males and young females at reproductive period in whole blood viscosity, and numerous studies previously showed that high hematocrit and blood viscosity were significantly correlated with male cerebrovascular disorders because of female menstruations, so there are significant gender differences in all viscosity parameters and hematocrit leading to lower blood viscosity in female [41].

Approximately 0.8% of total red blood cell reformed per day, and 80% of female erythrocytes were younger; this leads to lower erythrocyte rigidity in female in comparison with male and different studies illustrate that elevated blood viscosity increases the erythrocyte aggregation and inhibits erythrocyte deformability. Moreover, aged erythrocyte disturbed microcirculations and released hemoglobin from erythrocyte which cause nitric oxide depletion that leads to vasoconstriction and then decreases nitric oxide augment platelet activation and thrombosis, and this explained the lower levels of nitric oxide in male [42], so most of these studies coincide with our results which showed lower erythrocyte rigidity index in female in comparison with male; also the present study showed gender differences in therapeutics response toward vinpocetine and/or pyritinol.

Pyritinol improves blood viscosity via elevation of erythrocyte ATP which increases deformability and reduces the erythrocyte rigidity; thus acute high dose of pyritinol increases blood ATP in about 20%; also it increases erythrocyte cGMP, improves glucose metabolism, and augments acetylcholine-induced vasodilatation [43].

Therefore, the present study showed significant improvement in blood viscosity in addition to the amelioration of plasma viscosity which may be through ATP activation, but unfortunately level of ATP is not measured in this study due to limited facilities.

Erythrocytes enclosed considerable amounts of ATP formed via glycolysis pathway and in response to hypoxia, acidosis, and mechanical deformability, the erythrocytes release ATP sufficient for creation and stimulation of vascular endothelial purinergic receptors which induced nitric oxide and prostacyclin release causing vasodilation, but erythrocyte ATP efflux needs specific ion channels that are stimulated via pyritinol. Many studies showed that the erythrocyte participation in nitric oxide-dependent vasodilation improves tissue perfusions and decreases blood viscosity; this gives a new imminence for pathophysiology of blood viscosity disorders [44, 45].

Pyritinol like ascorbic acid is potent antioxidant and removes free radicals mainly hydroxyls radical which are generated during hydrogen peroxide and superoxide interactions; this hydroxyl radical damages erythrocyte membrane protein and cholesterol in addition to nucleic acid, so pyritinol protects erythrocyte membrane from oxidation, thus improving deformability and ameliorating RBC rigidity [46].

Moreover, pyritinol accelerates white blood cells and inflammatory cell migration into inflamed site without induction of inflammatory mediators releasing during acute and chronic inflammatory disorders associated with hyperviscosity like rheumatoid arthritis [47]. Also, triggered leucocytes increased blood viscosity via reduction in erythrocyte deformability and membrane lipid peroxidation; all these resulted from oxygen free radical, and because pyritinol is a potent scavenger it eliminates the effect of activated white blood cells on erythrocytes and thus on blood viscosity [48].

Erythrocytes are more vulnerable toward oxidative damage via free radicals due to higher hemoglobin and oxygen inside them and high lipid concentration in their membranes, so exposure to oxidative stress leads to erythrocyte rigidity, aggregation, and inhibition of deformability; therefore, oxidative stress is regarded as an important factor for elevation of blood viscosity [49], so the anti-inflammatory effects of pyritinol decrease the inflammatory proteins; therefore, it decreases plasma viscosity and improves the erythrocyte deformability; unfortunately, oxidative markers are not measured in this study.

Combined or joint effects of vinpocetine and pyritinol showed higher improvement in the blood viscosity because both agents are antioxidant like other potent antioxidants such as vitamin E, vitamin C, and other herbal extracts [50].

Plasma viscosity was regarded as marker of acute disease due to elevation of plasma protein; mainly fibrinogen also reflects the erythrocyte rigidity indirectly because erythrocyte rigidity index depends on plasma viscosity; only vinpocetine decreases fibrinogen level significantly, while pyritinol decreases plasma viscosity without affecting fibrinogen level; thrombocyte and leucocytes are not regarded as important factors for blood viscosity; moreover, blood viscosity is correlated with the shear stress, so higher shear stress prevents erythrocyte aggregations, but low shear stress increases their aggregations [51–53].

Additionally, in erythrocyte deformability the structural alterations were high and rapid at high shear blood viscosity compared to low shear due to erythrocyte viscoelasticity; therefore, vinpocetine and pyritinol enhance viscoelasticity through amelioration of low shear whole blood viscosity [54, 55].

The physiological response of increase 10% in hematocrit is elevation in blood viscosity by 20% resulting in reduction in blood flow and elevation of peripheral resistance leading to hypertension complications; the endothelia of atherosclerotic vessels lose their abilities for synthesis and releasing vasodilator nitric oxide, so the vasodilating effects of vinpocetine and pyritinol were capable of inducing vasodilation in elderly or long-term hypertension independent of nitric oxide, but they were capable of reducing blood pressure via reduction of whole blood viscosity, but the vasodilator leads to hypotension and collateral ischemia due to stasis of erythrocyte because of the capillary becoming much narrower for passage of erythrocytes. Therefore, reduction in blood viscosity is an optional way for reduction of blood pressure in complicated cerebrovascular disorders [56].

Therefore, dual combined or joint effects of pyritinol and vinpocetine produced significant rheological improvement via modulation of blood viscosity and other related hemorheological parameters.

## 5. Conclusions

Joint effects of vinpocetine and pyritinol improve blood and plasma viscosity in patients with cerebrovascular disorders and provide a new therapeutic model for prevention and progression of cerebrovascular disorders.

## Figures and Tables

**Figure 1:** Gender differences in RBS rigidity index (RRI) in responses to the vinpocetine and/or pyritinol.

**Table 1:** Rheological properties of oral vinpocetine 10 mg/day for two weeks in cerebrovascular disorders.

Variables	Before	After	*P* value
Hematocrit %	45.7 ± 0.23	44.2 ± 0.45	*P* > 0.05
Total serum protein g/dl	8.64 ± 0.21	8.15 ± 1.76	*P* > 0.05
Fibrinogen g/l	3.78 ± 0.87	2.01 ± 0.08	*P* < 0.05
Relative blood viscosity cP	4.33 ± 0.65	2.11 ± 0.03	*P* < 0.05
Actual blood viscosity cP	3.3685 ± 0.021	1.148 ± 0.032	*P* < 0.05
WBV-HSR cP	6.6009 ± 0.032	6.337 ± 0.011	*P* > 0.05
WBV-LSR cP	116.377 ± 0.165	97.935 ± 2.23	*P* < 0.01
RRI	2.17 ± 0.011	1.17 ± 0.087	*P* < 0.05
Plasma viscosity cP	1.55 ± 0.06	0.98 ± 0.08	*P* < 0.05
Kinematic viscosity	3.18 ± 0.17	1.083 ± 0.64	*P* < 0.05

WBV-HSR: whole blood viscosity high shear rate, WBV-LSR: whole blood viscosity low shear rate, and RRI: RBC rigidity index.

**Table 2:** Rheological properties of oral pyritinol 100 mg/day for two weeks in cerebrovascular disorders.

Variables	Before	After	*P* value
Hematocrit %	45.7 ± 0.23	45.6 ± 0.76	*P* > 0.05
Total serum protein g/dl	8.64 ± 0.21	8.55 ± 1.39	*P* > 0.05
Fibrinogen g/l	3.78 ± 0.87	3.65 ± 0.071	*P* > 0.05
Relative blood viscosity cP	4.33 ± 0.65	3.11 ± 0.29	*P* < 0.05
Actual blood viscosity cP	3.3685 ± 0.021	2.1485 ± 0.038	*P* < 0.05
WBV-HSR cP	6.6009 ± 0.032	5.472 ± 0.08	*P* > 0.05
WBV-LSR cP	116.377 ± 0.165	86.184 ± 0.032	*P* < 0.01
RRI	2.17 ± 0.011	2.17 ± 0.036	*P* > 0.05
Plasma viscosity cP	1.55 ± 0.06	0.99 ± 0.05	*P* < 0.05
Kinematic viscosity	3.18 ± 0.17	3.17 ± 0.07	*P* > 0.05

WBV-HSR: whole blood viscosity high shear rate, WBV-LSR: whole blood viscosity low shear rate, and RRI: RBC rigidity index.

**Table 3:** Dual combined effects of vinpocetine and pyritinol on hemorheological parameters in cerebrovascular disorders.

Variables	Before	After	*P* value
Hematocrit %	45.7 ± 0.23	43.1 ± 0.65	*P* < 0.05
Total serum protein g/dl	8.64 ± 0.21	8.12 ± 2.76	*P* > 0.05
Fibrinogen g/l	3.78 ± 0.87	1.99 ± 0.09	*P* < 0.05
Relative blood viscosity cP	4.33 ± 0.65	1.98 ± 0.02	*P* < 0.01
Actual blood viscosity cP	3.3685 ± 0.021	1.0185 ± 0.45	*P* < 0.05
WBV-HSR cP	6.6009 ± 0.032	5.172 ± 0.026	*P* > 0.05
WBV-LSR cP	116.377 ± 0.165	81.45918 ± 2.23	*P* < 0.01
RRI	2.17 ± 0.011	1.75 ± 0.03	*P* < 0.05
Plasma viscosity cP	1.55 ± 0.06	0.58 ± 0.006	*P* < 0.05
Kinematic viscosity	3.18 ± 0.17	0.960 ± 0.002	*P* < 0.01

WBV-HSR: whole blood viscosity high shear rate, WBV-LSR: whole blood viscosity low shear rate, and RRI: RBC rigidity index.
